# Mathematical Modeling and Numerical Simulation for the Outbreak of COVID-19 Involving Loss of Immunity and Quarantined Class

**DOI:** 10.1155/2022/3816492

**Published:** 2022-06-08

**Authors:** Faiza Arif, Zain Majeed, Jamshaid Ul Rahman, Naveed Iqbal, Jeevan Kafle

**Affiliations:** ^1^Abdus Salam School of Mathematical Sciences, Government College University, Lahore 54600, Pakistan; ^2^Department of Mathematics, College of Science, University of Ha'il, Ha'il 2440, Saudi Arabia; ^3^Central Department of Mathematics, Tribhuvan University Kirtipur, Kathmandu, Nepal

## Abstract

For the analysis of the recent deadly pandemic Sars-Cov-2, we constructed the mathematical model containing the whole population, partitioned into five different compartments, represented by SEIQR model. This current model especially contains the quarantined class and the factor of loss of immunity. Further, we discussed the stability of the SEIQR model (constructed on the basis of system of coupled differential equations). The basic reproduction that indicates the behavior of the disease is also estimated by the use of next-generation matrix method. Numerical simulation of this model is provided, the results are analyzed by theoretically strong numerical methods, and computationally known tool MATLAB Simulink is also used for visualization of the results. Validation of results by Simulink software and numerical methods shows that our model and adopted methodology are appropriate and accurate and could be used for further predictions on COVID-19. Our results suggest that the isolation of the active cases and strong immunization of patients or individuals play a major role to fight against the deadly Sars-Cov-2.

## 1. Introduction

At present, emergence of deadly respiratory virus COVID-19 throughout 209 countries of the world is a major global concern. Primarily, this virus was known as Severe Acute Respiratory Syndrome Coronavirus-2 (Sars-Cov-2), which initially came out in Wuhan city of China. COVID-19, which originated at the end of December 19 in Wuhan, China, is considered to be the third epidemic of CoV, and it is holding almost the same symptoms like Sars-CoV. And this disease is found to be more deadly than the coronavirus Sars.

Since its outbreak, this virus has caused enormous deaths up to 4,182,831 and has infected 195,345,791 people worldwide. The main cause of the outspread of this virus is the contact of infected person with healthy individuals because it was found in study that this infection is usually caused by transmission of globules through coughing or sneezing. These globules can stay in the air for a long time and can cause infection to others. However, it is quite challenging for the scientists to investigate the preventive measures under which the spread of this virus can be controlled and to produce a vaccination to fight against this virus. Until now, almost 13 vaccinations against this disease exist and scientists are still devoting their attentions to produce a strong vaccination against this virus. A huge amount of research has been carried out to look over the conditions and circumstances by which this deadly virus can be controlled. Scientists find out COVID-19 to be one of the crucial outbreaks that attack the respiratory system [1]. One of the main reasons behind the outspread of COVID-19 is due to the transmission of germs through respiratory globules among humans, and this virus is considered to be the vector transmission. the WHO (World Health Organization) warned that if control measures are not implemented in time, then the outbreak of the coronavirus can spread more rapidly [2].

Qualitative analysis using the concept of basic reproduction ratio estimated by next-generation matrix and stability theory of differential equations to examine the outburst of COVID-19 was studied by Olumuyiwa et al. [3]; basically, they estimated the epidemic behavior in Pakistan by using some previous statistical data from Pakistan and they applied numerical approaches Nsfd and Ode45 to figure out the study.

Researchers are adopting different tactics to investigate the growing behavior of the coronavirus and carrying out their studies to find out the ways to bring COVID-19 to an end. One of the methods of analyzing the behavior of diseases is compartmental modelling that is applicable to the mathematical models involving influential diseases. In this approach, the population is allocated to various compartments with particular labels, for example, susceptible (*S*) and infected (*I*). Mathematical models are quite helpful in investigating the behavior of viruses, diseases, or infections and help out to conclude under what circumstances the outbreaking virus can be eradicated or continued in citizens and are often useful in estimating the duration of an outbreak. These models are usually considered to take form of differential equations.

Annas et al. constructed the mathematical model to study the influential behavior of coronavirus [4, 5]; they also discussed the stability of their proposed model. Suleman et al., Ul Rahman et al., and Iqbal and Karaca numerically investigated the fractional model of HIV [6, 7, 8]. The National Health Organization instructed to keep away from infectious person or animals either with fever or any respiratory problems and also directed to wear surgical masks and directed continual use of hand sanitizers in public places for self-safety from infection. Social distancing or less crowded places can reduce the risk of spreading of coronavirus because it is more likely to spread in compact places. Batista constructed the SIR model to guess the finishing measurements of coronavirus [9]. Moreover, the basic reproductive number (*R*_0_) is very effective in approximating the transmission rate of an infection; i.e., it is also useful in estimating the ratio of occupants required to be immunized in order to wipe out the infection.

Basic reproductive number is estimated basically from the mathematical model, and in most epidemic models, the spreading rate of infection or disease-free equilibrium point is said to be endemic or stable if *R*_0_ lies between 0 and 1, otherwise it will be epidemic or unstable. Substantially, the larger the values of *R*_0_, the harder it is to take control of the outbreak of the disease. Zhao et al. proposed the test approximation of the basic reproductive number (*R*_0_) for the breakout of COVID-19 during its early stages [10, 11]. However, it is not that easy to find out the explicit expression for the basic reproductive ratio so more advanced approaches, e.g., next-generation matrix, are required to estimate the reproductive number [12]. The study of basic reproduction ratio (*R*_0_) for dissemination of epidemical infection was presented by Van den Driessche and Watmough, and they also bring forward the stability and unstability of infection free equilibrium based on reproductive ratio [13, 14].

The use of epidemic computational simulation models play a key role in estimating the transferal parameters and in guessing the influential behavior of the infection. These models are proven to be useful in depicting the growth rate or decay rate of viruses with the passage of time and are quite helpful in providing the control measures that can be adapted to reduce the spread of the disease. A lot of results and applications carried out from the simulation models of COVID-19 are being accepted and published. Abdulrahman presented the computer software Simulink program to track the contagious virus COVID-19. He used SEIRD and SIR epidemic models in the form of algebraic-differential equations and simulated the results by using Simulink approach [15].

One way of examining the influential growth of this deadly outbursts is to use the computer simulation block models. In various publications, different numerical as well as analytical approaches are taken into account to carry out the outputs of SIR, SEIR, and SEIRD models. A SIR model involving the immigration rate was proposed by Ud Din et al. They simulated their outputs by applying the approach of Nsfd and investigated the changing behavior of epidemic due to immigration factor between different classes [16].

Numerical approaches are also useful in analyzing the changing behavior of the outburst diseases and can provide some better precautionary measures to prevent the diseases transmission. In literature, average researchers have used meshless as well as numerical methods like FDM, FVM, FEM, Euler, and Runge-Kutta. But the classical numerical methods like RK and Euler are less computational, efficient, and easily applicable, as meshless methods are useful in simulating physical phenomena including biological as well as engineering-related problems, as if analyzed the SEIR model of disease by applying meshless methods like EFBMM and OSBMM [17].

Ahmed et al. adapted some numerical techniques, including Rk2, Rk4, and Euler's method as well as simulation process to study some mathematical models developed for COVID-19. Further, they estimated the epidemic size for Iraq and Turkey with the help of a logistic model [18, 19]. Maier and Brockmann presented the growth rate of COVID cases in contrast with the initial rate of suspected cases [20, 21]. Baba et al. numerically investigated the effects of the lockdown by constructing the model based on five equations and also discussed the equilibria and its stability [22, 23]. Zha et al. proposed the fuzzy-based approach in order to lessen the outbreak of the novel Sars-Cov-2 [24].

Bassetti et al. studied the contaminating behavior of COVID-19, and further, they investigated what obstacles we can face due to this virus [25, 26]. Cao et al. presented the study predicated on the Arimax and SEIR model; further, they proposed some precautionary measures to suppress COVID-19 [27, 28]. Chen et al. reported the Sars reappearance in COVID-19, and Diao et al. reported on the deletional behavior of T-cells because of Sars-Cov-2 [29, 30].

Peto, Hussain et al., and Kucharski et al. found in their study that people with less immunity are at risk of getting infectious; moreover, they suggested that this risk can be reduced if the population is tested weekly so that the infectious individual could be quarantined at time and the disease will be less likely to be spread and people can resume their normal life [31, 32, 33]. Tuli et al. suggested that machine learning is quite useful in finding what possible trajectory can a disease follow in the future. In order to trace the growing behavior of Sars-Cov-2, they proposed the model rest on machine learning [34]. Khoshnaw et al. pointed towards the significance of using computational simulation tools to forecast the behavior of infections. They bring forward the idea of sensitivity analysis to test the sensitivity of the models formulated on the basis of differential equations [35, 36].

Ul Rahman et al. proposed the model for paint industry effluent and simulated the results by using MATLAB Simulink tool [37].

The short-term analysis of Sars in three huge cities of India was investigated by Mandal et al.; also, they advanced the method to control out the basic reproduction ratio [38, 39]. Liu et al. studied the intercontinental tide of the respiratory Sars-Cov-2 [40, 41]. Neher et al. estimated how the discrepancy of seasonal forces helps in the modification of Sars-Cov-2 [42, 43]. Ozair et al. formulated the SIR model to study the transmission behavior of COVID-19 in Romania and Pakistan [44].

Egbetade et al. analyzed the SIR model of the infections and also discussed the existence of equilibria and the reaction of disease on the basis of *R*_0_ [45, 46]. Ul Rahman et al. used the concept of numerical simulation to model some industrial problems and analyzed the models by using numerical techniques and Simulink [47, 48]. Abdulrahman, Iqbal and Wu, and Rahim et al. used simulation programs to analyze the mathematical models constructed to study COVID-19 and biological models [49, 50, 51, 52].

From the above studies, it has been concluded that the reason behind the global outspread of COVID-19 is dense places and migration of infected people and loss of immunity in people to fight against diseases. Therefore, to control the outspread of CoV, it is necessary to quarantine the infected person and moreover, strong immunization of patients must be necessitated to get rid from this infection.

- In this study, we will estimate the control of some parameters including immunity parameter and isolation class that will be beneficial to provide some controlling features for the above-mentioned disease. This research work is constructed by the SEIQR model based on nonlinear differential equations, and the model is analyzed by the simulation block models and by using some numerical approaches. Furthermore, the stability of the reproduction ratio (*R*_0_) and the existence of disease-free equilibria are also studied. The idea of next-generation matrix is utilized to find out the reproduction ratio
- The summary of our work is as follows: we applied Euler's method, Rk4, and Ode45 to obtain the results for our differential-equation epidemic model
- Another aim is to estimate the local stability of reproductive number

For this purpose, we divided the paper in three sectors. The first section is for the mathematical model; in the second section, the stability analysis and the existence of equilibrium point are discussed; and in the last section, the numerical and graphical outcomes are represented.

The flow diagram of the SEIQR model is presented below. In the flow diagram (Figure 1), the transmission of population with different transition rates, among the five compartments, is shown. In Figure 1, the parameter *Z* is representing the rate of population joining the susceptible class and further, the individuals from the susceptible community are moving to the infected as well as exposed community with *β* force of infection. The parameter *πE* indicates the switching rate of individuals from the exposed to the infected class. The isolated class contains the individuals from the exposed and infected class, with *γ* and *σ* joining rates, respectively. Further, recovered individuals with lack of immunity leave the recovered class with *α* rate and move to the susceptible class.

## 2. Formulation of Mathematical Model

The SIR model is the simplest fundamental model constituting three compartments of complete population. And it was first used in 1916 and then in 1927 to estimate the behavior of diseases and viruses. Other models like SEIRD, SIRD, and SEIR are the extensions of this basic model.

The present model is the SEIQR model. As the reason behind the upsurge COVID-19 is the lack of immunity and the contact of infected patients with other healthy individuals, therefore, in the said work, the SEIQR stochastic mathematical model is formulated involving the immunity parameter and the quarantined community.

For this, the partition of whole population is placed in five different compartments named as (i) susceptible (*S*), (ii) exposed (*E*), (iii) infected (*I*), (iv) quarantined (*Q*), and (v) recovered (*R*).

The susceptible class contains those individuals having mild symptoms and who are at risk of getting infectious Table 1. The individuals who are needed to be quarantined are indulged in isolated class, and people who caught the disease are present in the infected class, whereas the recovered compartment contains those individuals who are either dead or have recovered from infection or the people who are still at risk of getting infectious again due to less immunity.

### 2.1. SEIQR Mathematical Model

The SEIQR model is given by the following nonlinear 1st-order differential equations, and the description of each compartment is given Table 1.

(1) $$\begin{array}{c} \frac{dS\left(t\right)}{dt}=Z-\mu S\left(t\right)-\beta \left(N\right)S\left(t\right)\left(E\left(t\right)+I\left(t\right)\right)+\alpha R\left(t\right),\\ \frac{dE\left(t\right)}{dt}=\beta \left(N\right)S\left(t\right)\left(E\left(t\right)+I\left(t\right)\right)-\pi E\left(t\right)-\left(\mu +\gamma \right)E\left(t\right),\\ \frac{dI\left(t\right)}{dt}=\pi E\left(t\right)-\mu I\left(t\right)-\sigma I\left(t\right),\\ \frac{dQ\left(t\right)}{dt}=\gamma E\left(t\right)+\sigma I\left(t\right)-\theta Q\left(t\right)-\mu Q\left(t\right),\\ \frac{dR\left(t\right)}{dt}=\theta Q\left(t\right)-\mu R\left(t\right)-\alpha R\left(t\right). \end{array}$$

Each equation is describing the transmission behavior of individuals in the respective compartments. By this transmission, number of individuals can vary in each of the five compartments. The description of the transition rates in each cell is given in Table 2.

Let us define the initial conditions to be *S*(0) = *S*_0_ ≥ 0, *E*(0) = *E*_0_ ≥ 0, *I*(0) = *I*_0_ ≥ 0, *Q*(0) = *Q*_0_ ≥ 0, and *R*(0) = *R*_0_ ≥ 0.

The precise definition of the compartments used in the formulation of the model can be seen from Table 1 [3, 53, 54].

## 3. Positivity and Stability of Solution

### 3.1. For Positivity and Boundedness of Solution

For the positiveness of the solution and bounded solution of the above system, it is necessary that the solution maintains nonnegativity for all *t* ≥ 0.

And it was found that

(2) $$\begin{array}{c} \frac{dS\left(t\right)}{dt}=\mu \geq 0\;\text{at }S=0,\\ \frac{dE\left(t\right)}{dt}=\beta NSI\geq 0\;\text{at }E=0,\\ \frac{dI\left(t\right)}{dt}=\pi E\left(t\right)\geq 0\;\text{a}t\;I=0\\ \frac{dQ\left(t\right)}{dt}=\gamma E\left(t\right)+\sigma I\left(t\right)\geq 0\;\text{at }Q=0,\\ \frac{dR\left(t\right)}{dt}=\theta Q\left(t\right)\geq 0\;\text{at }R=0. \end{array}$$

The interpretation of the parameters used in the formulation of the model can be seen from Table 2 given below.

### 3.2. Stability of Solution and State of Existence of Positive Equilibrium Point

The stability of our mathematical model mainly relies on the basic reproduction ratio; moreover, the existence of positive equilibria is also depending on *R*_0_. To determine *R*_0_, we used the next-generation matrix method and obtained

(3) $$\begin{array}{c} R_{0}=\beta N\frac{\mu +\pi +\sigma }{\left(\sigma +\mu \right)\left(\pi +\gamma +\mu \right)}, \end{array}$$

since *R*_0_ is defined by the relation

(4) $$\begin{array}{c} R_{0}=\rho \left(FV^{-1}\right). \end{array}$$

*R*_0_ equals the eigenvalue of *FV*^−1^, where *F* includes the terms with secondary infectious disease and *V* includes the terms other than the secondary infectious disease.

And the stability of system can be decided from *R*_0_, i.e.,

- the proposed system is stable with infection-free equilibria for *R*_0_ < 1
- the proposed system is unstable with infectious equilibria for *R*_0_ > 1

The stability discussed here is basically local stability.

### 3.3. Simulink Block Model

In order to speculate and trace the eruption of Sars-Cov-2, we proffered the computer-based simulation scheme in this considered article. For this objective, the respective differential equations are simulated with the help of blocks available in the library browser of Simulink-MATLAB. Simulink tool is easy to use for the purpose of predicting behavior of any natural phenomenon or system. The above considered mathematical model is rooted in Simulink with the help of block diagram given in the appendix.

## 4. Numerical Simulation and Results

For the output of the present model, we implemented two numerical methods Euler's method and Rk4. Also, we simulated our results with the help of simulation by using Simulink blocks.

The dynamical behavior of population in all five classes is shown graphically by taking different time periods. Further, the comparison of three methods Ode45/Simulink, Rk4, and Euler method is shown in graphs.

The changing behavior of population in various compartments for the stable infection, i.e., for endemic case *R*_0_ < 1.

Dynamics of population over 365 days, in various compartments for unstable infection, i.e., for pandemic case *R*_0_ < 1.

As no proper vaccination for the disease is discovered yet, so the entire individuals are at risk of getting contaminate by this infection. That is why the whole population is often put into the susceptible class. From the susceptible class, the entities of that class can get infected by making contact with an infectious person and then, they can join the infected class as well as the exposed class. The differential behavior of the susceptible entities is shown in Figure 2(a) for the case of endemic disease. In Figure 2(a), the behavior is depicted over the period of 20 days as one can see that when we have an endemic case, so the susceptible class has a constant rate of variation as people are at less risk of getting engaged to the disease and there will be less movement of individuals from this class to other compartments. Moreover, in Figure 2(b), the graph is depicting the changing behavior of the population in the susceptible class over the period of 40 days and in Figures 3(a) and 3(b), the variation in susceptible individuals is shown over the period of 60 and 80 days, respectively. Another aspect of the constant variation of individuals in the susceptible class is that when we have the population with strong immunity system, i.e., less people will get infected to the disease. The above-mentioned graphs are drawn for the strong immunity parameter. And all these results are carried out with the help of Ode45, Rk4, and Euler's method.

In Figures 4(a) and 4(b), the transition behavior of the population having less immunity is discussed, since for less immunization factor, there is higher probability of getting involved with the infection. As one can see from both graphs, individuals from the susceptible cell are becoming part of infected as well as exposed cells. The decreasing behavior is depicting the tendency of people getting infectious and exposed.

The variation of entities in the exposed cell considering the case of endemic virus is depicted in Figures 5(a), 5(b), 6(a), and 6(b). One can see that the graph of this class is illustrating the sharp reduction throughout different periods of time. The reason behind this decrement is the immigration of individuals from the exposed class to the infected class. As the exposed individuals have almost 60% signs of the disease, so they are almost considered to be infected and therefore, the graphs are showing the sharp rate of variation from the exposed cell to the infected one.

The evolution of individuals in the infected community is portrayed in Figures 7 and 8. The transition behavior of individuals in the infected class is depicted in Figure 7(a) over the period of 20 days; the initial increment is due to the joining of the infected cell of exposed people, and in Figure 7(b), the graph is drawn for the time period of 40 days; the early increasing behavior is due to the increase of population in the infected cell, and the decreasing behavior later is due to the movement of patients from the infected to the quarantined cell. In Figures 8(a) and 8(b), the dynamical behavior of the population is illustrated over the period of 60 and 80 days, respectively. The diminution after some time is due to the immigration of patients to the isolated cell.

As we are considering the isolation of patients in order to prevent the further spread of the disease, so the infected patients are needed to be quarantined for the reduction of the spread. The dynamical behavior of the quarantined population is shown in Figures 9 and 10 for different time periods. From these graphs, it can be seen that people are getting involved in the recovered cell with sharp rate if they are quarantined in time. The variation of recovered population is drafted in Figures 11 and 12; it can be seen that the graphs are depicting an increasing behavior; the reason behind this sharp recovery is due to the isolation of infected individuals and the strong immunization of the patients. The initial decrement is due to the less immunity factors and the deaths of patients either by disease or other reasons.

The dynamics of population in the susceptible class is shown in Figures 13(a) and 13(b); in Figure 13(a); the behavior is shown for the strong immunity parameter; on the other hand, the graphical results are depicted by considering weak immunity among individuals. In Figure 14(a), transition behavior in the exposed class is depicted over 365 days; the decreasing effect is due to the transition rate of individuals from the exposed class to the infected class, in which in Figure 14(b), the dynamics of population in the isolated class displays the initial increment and then decrement of population; this fluctuation is due to the joining and motion of individuals in this class from other classes. In Figure 14(c), the dynamics of individuals shows the rise in population of the isolated class and the later declining behavior shows the flow population from the isolated class to the recovered class. Further, in Figures 15(a) and 15(b), the weak and strong immunity among individuals is considered, respectively; Figure 15(a) shows a slow rate of recovery due to loss of immunity; and Figure 15(b) shows a sharp rate of recovery due to strong immunity.

Now, the illustration for the transmission dynamics of population in each compartment is considered for the case of epidemic disease. In Figures 16(a) and 16(b), the rate of change of population in the susceptible class is illustrated for 20 and 40 days, respectively, by taking into account the epidemic behavior of disease. We can see the suppressed behavior of population in the *S* class that is due to the fact that people from this class can catch the infection and can move to other compartments. In the endemic case, we have a higher rate of transition from one cell to another, as compared to the epidemic case. The same reaction of population is shown in Figures 17(a) and 17(b) considering 60 days and 80 days, respectively.

In Figures 18 and 19, transmission dynamics of population in the exposed cell is given. The prime rise is by the increase in population of this cell, as from the susceptible class, more individuals are engaging in this class and the later decrease is due to the fact of epidemic behavior, as disease is not in control so exposed individuals are getting involved in infected cell. And the reason behind the inflation of population in the infected class is the excessive amount of indulgence of individuals between the exposed and infected classes due to the epidemic behavior as one can see in Figures 20 and 21.

Figures 22 and 23 show the dynamics of population in the isolated compartment over 20, 40, 60, and 80 days, respectively. The recovered rate of the population is presented in Figures 24 and 25; it can be seen from the graphs that in the case of epidemic virus, we have slow-going recovery of infected individuals as compared to those in the case of endemic behavior. Similarly, the dynamical behavior of the population over 365 days is given in Figures 26, 27, and 28 for each cell. It is readily apparent from the graphical results that

- for

(5) $$\begin{array}{c} R_{0}=\beta N\frac{\mu +\pi +\sigma }{\left(\sigma +\mu \right)\left(\pi +\gamma +\mu \right)}<1, \end{array}$$

the virus is endemic and stable so less people will catch the infection

(ii) for

(6) $$\begin{array}{c} R_{0}=\beta N\frac{\mu +\pi +\sigma }{\left(\sigma +\mu \right)\left(\pi +\gamma +\mu \right)}>1, \end{array}$$

the virus is epidemic and unstable so, more people will catch the infection

The changing behavior of population in various compartments for unstable infection, i.e., for pandemic case *R*_0_ > 1.

Dynamics of population over 365 days, in various compartments for unstable infection, i.e., for pandemic case *R*_0_ > 1.

## 5. Conclusion

In the said study, we concluded that isolation of the infected person and strong-immunization of the individuals can be taken as precautionary measures to control the virus. By following the Sops implemented by the government, we can prevent the further outbreak of this disease. For the unstable case, it can be seen that there is sharp variation of entities among all five classes. And for the lower immunity factor, individuals are still at risk of getting infectious and there are fewer chances of recovery. And for the stable case, it is apparent from graphical results that less people are exposed to infection. As in the susceptible class, we have constant behavior of population with zero loss-immunity parameter. But if we include the lack of immunity parameter, we can see that more people are joining the exposed and isolation classes but the situation is in control since we have endemic behavior here. In Section 3, it is discussed in detail. The comparison of the three methods can also be seen from the graphs. It can be seen that Ode45 is more accurate than Euler's method (1st-order RK method) and Rk4 as it is built in MATLAB and it implements Rk4 or Rk5 to solve the equations.

Validation of results by Simulink software and numerical methods shows that our model and adopted methodology are appropriate and accurate and could be used for further predictions on COVID-19.

## Figures and Tables

**Figure 1:** Flowchart of the proposed SEIQR model.

**Figure 2:** Dynamical behavior of population in the susceptible compartment with strong immunity.

**Figure 3:** Dynamical behavior of population in the susceptible compartment with strong immunity.

**Figure 4:** Dynamical behavior of population in the susceptible compartment with less immunity.

**Figure 5:** Dynamical behavior of population in the exposed compartment.

**Figure 6:** Dynamical behavior of population in the exposed compartment.

**Figure 7:** Dynamical behavior of population in the infected compartment.

**Figure 8:** Dynamical behavior of population in the infected compartment.

**Figure 9:** Dynamical behavior of population in the isolated compartment.

**Figure 10:** Dynamical behavior of population in the isolated compartment.

**Figure 11:** Dynamical behavior of population in the recovered compartment.

**Figure 12:** Dynamical behavior of population in the recovered compartment.

**Figure 13:** Dynamical behavior of population in the susceptible compartment.

**Figure 14:** Dynamics of population in exposed, infected, and isolated compartments.

**Figure 15:** Dynamical behavior of population in the recovered compartment.

**Figure 16:** Dynamical behavior of population in the susceptible compartment.

**Figure 17:** Dynamical behavior of population in the susceptible compartment.

**Figure 18:** Dynamical behavior of population in the exposed compartment.

**Figure 19:** Dynamical behavior of population in the exposed compartment.

**Figure 20:** Dynamical behavior of population in the infected compartment.

**Figure 21:** Dynamical behavior of population in the infected compartment.

**Figure 22:** Dynamical behavior of population in the isolated compartment.

**Figure 23:** Dynamical behavior of population in the isolated compartment.

**Figure 24:** Dynamical behavior of population in the recovered compartment.

**Figure 25:** Dynamical behavior of population in the recovered compartment.

**Figure 26:** Dynamics of population in susceptible and exposed compartments.

**Figure 27:** Dynamical behavior of population in infected and quarantined compartments.

**Figure 28:** Dynamical behavior of population in recovered compartment.

**Figure 29:** Simulink block model diagram of the considered SEIQR mathematical model.

**Table 1:** Definition of the compartments.

Compartments	Brief definition
*S*	Susceptible community (susceptible to disease)
*E*	Exposed community (those people who come in contact with the virus)
*I*	Infected community (when someone is exposed to the disease and having 70% symptoms)
*Q*	Quarantined community
*R*	Recovered community

**Table 2:** Precise interpretation of the parameters.

Parameters	Interpretation
*Z*	Rate of individuals joining susceptible class
*μ*	Defining death toll due to virus and by natural means
*β*	Rate of susceptible individuals joining exposed and infected individual class
*α*	Lack of immunity toll
*π*	Exposed class joining infected individuals
*γ*	Immigration rate of exposed individuals to quarantined class
*σ*	Rate at which infected individuals are joining quarantined class
*θ*	Recovery rate of quarantined population

## Data Availability

The numerical data used to support the findings of this study are included within the article.

## Appendix

### A. Simulink Block Diagram

Simulink software is helpful to analyze the performance of any system or reaction of any natural phenomenon. Simulink tool is quite handy for the prediction and forecasting of any disease or infection. This tool is based on block diagrams and is beneficial in modeling and investigating the dynamical behavior of various phenomena. Engineers and scientists use Simulink software to test their proposed designs and models before finalizing their results. A mathematical model (constructed with the help of block diagrams) is required to start up the simulation program.

It is available in the main page of MATLAB. One can click on the Simulink icon, and it opens up with the Simulink start page. There, it appears with Simulink library browser constituting a huge library of blocks like math operations, sinks, sources, and commonly used blocks. The above mathematical model presented in Figure 29 is simulated by the formulation of block models based on integrators, gains, add blocks, product, and scope.

The product, integrator, sum, gain, and scope are available in the commonly used block library but they have different libraries too. The add and gain block is also available in the library of math operations; display and scope can be found in sinks. The add block is used to sum the inputs, the product block is used the multiply the inputs, and scope represents the results graphically. And integrator is accessible from continuous block library. The integrator block integrates the input signal with respect to time.

The outputs for the presented formulated model was simulated with the help of computer simulation software which solves the models with the help of block diagrams. The Simulink model is given by the following figure.

## Additional Points

*Highlights*. The SEIRQ model is modified to study the epidemic Sars-Cov-2. The problem is analyzed by MATLAB Simulink software and numerical methods (Euler method) and (*Rk*4). Evaluation of basic reproductive number is done by the next-generation matrix method. Local stability of infection-free equilibria is discussed. Numerical simulation is performed for each class considered in the modified SEIQR model. Results obtained for each class considering epidemic and endemic behavior of disease are represented graphically

## References

[1] Hoehl S., Rabenau H., Annemarie B. (2020). Evidence of SARS-CoV-2 infection in returning travelers from Wuhan, China. *New England Journal of Medicine*.

[2] Wai-Kit M., Huang J., Zhang C. J. P. (2020). *Breaking down of the healthcare system: mathematical modelling for controlling the novel coronavirus (2019-nCoV) outbreak in Wuhan, China*.

[3] Olumuyiwa J. P., Qureshi S., Yusuf A., Al-Shomrani M., AbioyeIdowu A. (2021). A new mathematical model of COVID-19 using real data from Pakistan. *Results in Physics*.

[4] Annas S., Pratama M. I., Rifandi M., Sanusi W. (2020). Stability analysis and numerical simulation of SEIR model for pandemic COVID-19 spread in Indonesia. *Chaos, Solitons & Fractals*.

[5] Ndaïrou F., Area I., Nieto J. J., Torres D. F. (2020). Corrigendum to "Mathematical modeling of COVID-19 transmission dynamics with a case study of Wuhan" [Chaos Solitons Fractals 135 (2020), 109846]. *Chaos, Solitons and Fractals*.

[6] Suleman M., Lu D., He J. H., Farooq U., Hui Y. S., Rahman J. U. (2018). Numerical investigation of fractional HIV model using Elzaki projected differential transform method. *Fractals*.

[7] Ul Rahman J., Lu D., Suleman M., He J. H., Ramzan M. (2019). He-Elzaki method for spatial diffusion of biological population. *Fractals*.

[8] Iqbal N., Karaca Y. (2021). Complex fractional-order HIV diffusion model based on amplitude equations with Turing patterns and Turing instability. *Fractals*.

[9] Batista J. (2020). *Estimation of the final size of the coronavirus epidemic by SIR model*.

[10] Zhao S., Lin Q., Ran J. (2020). Preliminary estimation of the basic reproduction number of novel coronavirus (2019-nCoV) in China, from 2019 to 2020: A data-driven analysis in the early phase of the outbreak. *International journal of infectious diseases*.

[11] Chen T. M., Rui J., Wang Q. P., Zhao Z. Y., Cui J. A., Yin L. (2020). A mathematical model for simulating the phase-based transmissibility of a novel coronavirus. *Infectious Diseases of Poverty*.

[12] Pauline V. D., Watmough J. (2008). Further notes on the basic reproduction number. *Mathematical epidemiology*.

[13] Pauline V. D., Watmough J. (2002). Reproduction numbers and sub-threshold endemic equilibria for compartmental models of disease transmission. *Mathematical Biosciences*.

[14] Liu Y., Gayle A. A., Wilder-Smith A., Rocklöv J. (2020). The reproductive number of COVID-19 is higher compared to SARS coronavirus. *Journal of travel medicine*.

[15] Ismael A. (2020). SimCOVID: an open-source simulation program for the COVID-19 outbreak.

[16] Din R. U., Shah K., Ahmad I., Abdeljawad T. (2020). Study of transmission dynamics of novel COVID-19 by using mathematical model. *Advances in Difference Equations*.

[17] Asif M., Ali Khan Z., Haider N., al-Mdallal Q. (2020). Numerical simulation for solution of SEIR models by meshless and finite difference methods. *Chaos, Solitons Fractals*.

[18] Ayub A., Salam B., Mohammad M., Akgul A., Khoshnaw S. H. A. (2020). Analysis coronavirus disease (COVID-19) model using numerical approaches and logistic model. *AIMS Bioengineering*.

[19] Nesteruk I. (2020). *Statistics based predictions of coronavirus 2019-nCoV spreading in mainland China*.

[20] Benjamin F. M., Brockmann D. (2020). Effective containment explains subexponential growth in recent confirmed COVID-19 cases in China. *Science*.

[21] Sarinya K., Humphries U., Khan A., Yusuf A. (2021). Model of rice blast disease under tropical climate conditions. *Chaos, Solitons & Fractals*.

[22] Baba I. A., Yusuf A., Nisar K. S., Abdel-Aty A. H., Nofal T. A. (2021). Mathematical model to assess the imposition of lockdown during COVID-19 pandemic. *Results in Physics*.

[23] Anastassopoulou C., Russo L., Tsakris A., Siettos C. (2020). Data-based analysis, modelling and forecasting of the COVID-19 outbreak. *PLoS One*.

[24] Zha T. H., Castillo O., Jahanshahi H., Yusuf A., Alsaadi F. E. (2021). A fuzzy-based strategy to suppress the novel coronavirus (2019-NCOV) massive outbreak. *Applied and Computational Mathematics*.

[25] Matteo B., Vena A., Giacobbe D. R. (2020). The novel Chinese coronavirus (2019-nCoV) infections: challenges for fighting the storm. *Euorpean Journal of Clinical Investigation*.

[26] Rothan H. A., Byrareddy S. N. (2020). The epidemiology and pathogenesis of coronavirus disease (COVID-19) outbreak. *Journal of autoimmunity*.

[27] Cao J., Jiang X., Zhao B. (2020). Mathematical modeling and epidemic prediction of COVID-19 and its significance to epidemic prevention and control measures. *Journal of Biomedical Research & Innovation*.

[28] Nishiura H., Linton N. M., Akhmetzhanov A. R. (2020). Serial interval of novel coronavirus (COVID-19) infections. *International Journal of Infectious Diseases*.

[29] Chen D., Lei X. W., Huang Z., Liu Z., Gao J., Peng L. (2020). Recurrence of positive SARS-CoV-2 RNA in COVID-19: a case report. *International Journal of Infectious Diseases*.

[30] Diao B., Wang C., Tan Y. (2020). Reduction and functional exhaustion of T cells in patients with coronavirus disease 2019 (COVID-19). *Frontiers in Immunology*.

[31] Peto J. (2020). Covid-19 mass testing facilities could end the epidemic rapidly. *BMJ*.

[32] Hussain S., Madi E. N., Iqbal N., Botmart T., Karaca Y., Mohammed W. W. (2021). Fractional dynamics of vector-borne infection with sexual transmission rate and vaccination. *Mathematics*.

[33] Kucharski A. J., Russell T. W., Diamond C. (2020). Early dynamics of transmission and control of COVID-19: a mathematical modelling study. *Infectious diseases*.

[34] Tuli S., Tuli R., Gill S. S. (2020). Predicting the growth and trend of COVID-19 pandemic using machine learning and cloud computing. *Internet of Things*.

[35] Khoshnaw S. H., Salih R. H., Sulaimany S. (2020). Mathematical modelling for coronavirus disease (COVID-19) in predicting future behaviours and sensitivity analysis. *Mathematical Modelling of Natural Phenomena*.

[36] Tang B., Wang X., Li Q. (2020). Estimation of the transmission risk of the 2019-nCoV and its implication for public health interventions. *Journal of Clinical Medicine*.

[37] ul Rahman J., Mohyuddin M. R., Satyanarayana S. V., Zahoor S., Al-Ghareebi A. (2016). Mathematical and Simulink model for paint industry effluent. *DJ Journal of Engineering Chemistry and Fuel*.

[38] Mandal M., Jana S., Nandi S. K., Khatua A., Adak S., Kar T. K. (2020). A model based study on the dynamics of COVID-19: prediction and control. *Chaos, Solitons & Fractals*.

[39] Rahman B., Aziz I. A., Khdhr F. W., Mahmood D. F. (2020). Preliminary estimation of the basic reproduction number of SARS-CoV-2 in the Middle East. *Bull World Health Organ*.

[40] Liu Q., Liu Z., Zhu J. (2020). *Assessing the global tendency of COVID-19 outbreak*.

[41] Atangana A. (2020). Modelling the spread of COVID-19 with new fractal-fractional operators: can the lockdown save mankind before vaccination?. *Chaos Solitons Fractals*.

[42] Neher R. A., Dyrdak R., Druelle V., Hodcroft E. B., Albert J. (2020). Potential impact of seasonal forcing on a SARS-CoV-2 pandemic. *Swiss medical weekly*.

[43] Hui David S., Azhar I., Madani T. A. (2020). The continuing 2019-nCoV epidemic threat of novel coronaviruses to global health -- the latest 2019 novel coronavirus outbreak in Wuhan, China. *International Journal of Infectious Diseases*.

[44] Ozair M., Hussain T., Hussain M., Awan A. U., Baleanu D., Ali Abro K. (2020). A mathematical and statistical estimation of potential transmission and severity of COVID-19: a combined study of Romania and Pakistan. *BioMed Research International*.

[45] Egbetade S. A., Salawu I. A., Fasanmade P. A. (2018). Local stability of equilibrium points of a SIR mathematical model of infectious diseases. *World Journal of Research and Review*.

[46] Hyun M. Y. (2014). The basic reproduction number obtained from Jacobian and next generation matrices - a case study of dengue transmission modelling. *Biosystems*.

[47] Rahman J. U., Khan U., Ahmad S. (2019). Numerical simulation of Darcy-Forchheimer 3D unsteady nanofluid flow comprising carbon nanotubes with Cattaneo-Christov heat flux and velocity and thermal slip conditions. *Processes*.

[48] ul Rahman J., Mohyuddin M. R., Anjum N., Zahoor S. (2015). Mathematical modelling & simulation of mixing of salt in 3- interconnected tanks. *Journal of Advances in Civil Engineering*.

[49] Abdulrahman I. (2020). *SimCOVID: open-source simulation programs for the COVID-19 outbreak*.

[50] Iqbal N., Wu R. (2019). Pattern formation by fractional cross-diffusion in a predator-prey model with Beddington-DeAngelis type functional response. *International Journal of Modern Physics B*.

[51] Iqbal N., Wu R. (2019). Motifs de Turing induits par reaction-diffusion croisee dans un systeme bidimensionnel avec un effet Allee fort. *Comptes Rendus Mathematique*.

[52] Rahim H., Iqbal N., Cong C., Ding Z. (2019). Pattern selection of three components Gray-Scott model. *Journal of Physics: Conference Series*.

[53] Ng K. Y., Gui M. M. (2020). COVID-19: development of a robust mathematical model and simulation package with consideration for ageing population and time delay for control action and resusceptibility. *Physica D: Nonlinear Phenomena*.

[54] Youssef H., Alghamdi N., Ezzat M. A., el-Bary A. A., Shawky A. M. (2021). Study on the SEIQR model and applying the epidemiological rates of COVID-19 epidemic spread in Saudi Arabia. *Infectious Disease Modelling*.

